RETRACTED

# Font Design in Visual Communication Design of Genetic Algorithm

**DOI:** 10.1155/2022/6897115

**Published:** 2022-06-07

**Authors:** Yue Wang, Won-jun Chung

**Affiliations:** ^1^Department of Visual Design, School of Architecture and Design, Dongmyong University, Busan 48520, Republic of Korea; ^2^Department of Advertising, College of Media, Linyi University, Linyi 276000, Shandong, China

## Abstract

The text has played an essential role in the advancement of human civilization. It is used now as a valuable cultural heritage that has been experienced for a thousand years. The passing text must have its irreplaceable advantages and charm. People are extremely sensitive to visual symbols, and it is also the first step in which people can know things. Most of the books in today's market focus on pictures and colors, which ignores the design of the text. This makes the text boring taste, causing the reader's visual fatigue, which is not conducive to readers absorbing information through books. Therefore, this paper studies the font design in the design of the visual algorithm based on the genetic algorithm, and the font design is analyzed by the particle swarming algorithm, the decision MIMO-SCMA system of the genetic algorithm. It aims to address the dryness of today's texts by constructing texts that are instantly recognizable and visually appealing to readers. Through innovative visual concepts, readers can enjoy the process of acquiring knowledge. In this paper, to investigate the effectiveness of the genetic algorithm in font design, the number of experimental research subjects was set to 300, and 280 valid questionnaires were collected to investigate the satisfaction of users with the newly designed fonts. Experiments showed that the visual communication design based on a genetic algorithm has increased by 6.52% for the design satisfaction and the number of fonts that use the system is also increasing.

## 1. Introduction

The text is a set of visual symbols, transformed from writing into a specific text, which is the value given to the text. The text is an important part of the information transfer, as an image color is an important visual element. In the context of visual communication, the visual meaning of “font” is personal. Whether it is e-mail, books, brochures, websites, and magazines, these designs have no difference in text. However, so far, the design and structure of “font” have been ignored. The genetic algorithm introduced in font design in visual communication design can make the font design provide valuable information to deep visual communication memory. In the development and design of the font, it integrates new features, making the creative design of the fonts widely spread, which has great significance for the development of the text.

RETRACTED

With the development of intelligent terminals, the Internet of Things, the application of genetic algorithms is increasingly popular, and many teams are excavating and researching. Wenskovitch et al. explored the concept of using artificial intelligence factors in programming languages. He modeled the learning behavior of the adapter group and related rational factors in the financial system. The relationship between code encoding and genetic algorithm integration properties is described in detail [1]. Chun proposed a new method for improving power generation system maintenance. The proposed method uses the genetic algorithm to achieve the optimal solution to the annual Lole value of the energy system during analysis [2]. Zhou et al. used the genetic algorithm to diagnose cardiovascular disease and to increase its initial density, which provides the optimum density for neural networks, increasing the efficiency of neural networks by about 10% [3]. Devornique et al. recommended optimizing the linear and longitudinal alignment of the *U* model. Digital samples are provided to compare the proposed technology with available methods, whose results prove the high efficiency of the proposed algorithm [4]. For multicenter optimization issues, Mercado-Borrayo et al. proposed a genetic algorithm to effectively solve these problems [5]. Xie et al. are testing a new hybrid calculation model in predicting future natural gas demand. They proposed a model binding on a genetic algorithm (GA) and other methods to construct a natural oil pipeline distribution model [6]. Wang proposed a new method based on static reactive energy recovery and traditional power system stability. This method is based on the connection between the genetic algorithm (GA) and the rough set process. What he proposed is designed to reduce the calculation time and reduce the storage capacity required for optimization and improve the performance stability of the power system [7]. From the above study, the current font design problems can be seen: first, the font is too monotonous compared to the picture, which cannot attract the reader's attention; second, the design of the font is about the transmission of culture, a single font form, which is not conducive to the transmission of colorful culture. Based on the above problems, this paper will focus on the analysis of font design to facilitate the inheritance and development of culture.

Visual communication is a communication service using a visual language, that is, a visual aid, which delivers information through optical media. Dawid and Kopel, to create a more beautiful graffiti, combined cloud computing and the Internet of Things, providing more visual communication elements. This provided resources for creators, which is a continuous creation enthusiasm [8]. Volkanovski et al. completed training through a visual exchange, providing the first algorithm for visual and social understanding of how to cooperate to support text processing to support visual exchange [9]. Zeinab et al. introduced signal flexibility to explain signal differences in different receivers and environments. Media reports are signals that accumulate from stock trading to games. Signal and visual kisses are used to affect funding decisions [10]. Alavidoost et al. determined many different stages of auditory interaction based on different time functions that affect the reaction of the audiovisual process (only affecting the auditory and audiovisual processes). It provided a unique way to explore acoustic interactions and measure the demand in short-term acoustic applications [11]. For multicenter optimization issues, Gong et al. and others proposed a genetic algorithm to effectively solve these problems [12]. Panapakidis and Dagoumas were testing a new hybrid calculation model in predicting future natural gas demand. They used their proposed model to construct a natural oil pipeline distribution model [13]. Fetouht Zakyms proposed a new method based on static reactive energy recovery and traditional power system stability. This method is based on the connection between the genetic algorithm (GA) and the rough set process. The proposed method is intended to reduce the calculation time and reduce the storage capacity required for optimization and improve the performance stability of the power system [14]. These studies have shown that genetic algorithms have been widely used in people's lives.

RETRACTED

The font is the charm after the evolution of history and culture, which is the basis of cultural development and inheritance. It promotes not only the development of culture but also the enjoyment of readers' visual aesthetics. Based on the development of the state design, this paper analyzes the readers by using the genetic algorithm and transmits text through visual communication systems. In this study, under the support of the genetic algorithm, the fonts were designed in this article for reader and text development. In this paper, we will combine genetic algorithms to design fonts and change the problems in the evolution of fonts nowadays, to attract users to increase their usage of fonts and increase their satisfaction.

The font is the charm of historical and cultural evolution and is the basis of cultural development and transmission. It not only promotes the development of culture but also is a visual and aesthetic enjoyment for readers. However, due to the general neglect of the majority of people nowadays, there is a serious impact on the development of fonts. Based on the development of font design nowadays, this paper influences the development of the text by using genetic algorithms, visual communication design to analyze the psychology of readers, and design fonts that are more acceptable to readers.

This article has an innovative point as follows:

1. In this paper, the genetic algorithm was introduced in the font design, analyzes the reader's psychology through a genetic algorithm, and designed the font that satisfies readers
2. This paper proposed an information platform for professionalism, openness, and practical construction for visual communication design
3. This article will also analyze the export methods and standard laws of words and then guide the application in modern design

## 2. Construction Based on the Visual Communication System

### 2.1. Relationship Chain in Visual Communication

Like the process of information visualization, visual conveyors ultimately help companies create value. Although there are many design categories and specific links, it is easy to customize business links. This article carefully develops internal visual conveying procedures by content and type, that is, from the outside: visual creativity, visual synthesis, process, control, and link. With the “external impact” as the main category, it encloses all external factors that affect the performance of the visual conveying process from different angles, which master the communication status of the internal and external communication links [15].

### 2.2. Value Link

In this article, based on economic-related theoretical boundary conditions, the value chain is only narrowly defined as a value chain produced by a series of value-added processes such as research, design, production, and marketing. Visual conveying is a circulation communication in the value chain. It is an intermediate link in the value chain, interacts with other links, and is affected by a wide range of business and social foundations.

As shown in Figure 1, the “value chain link” during visual conveying is a process management process and integrated creativity that promotes visual communication. Absorbing and assimilating the background of the era, and based on the understanding of the work itself, the field of visual communication affects the performance of artistic creation. During the further process of visual conveying processes, the production process must be checked and calibrated again and again to make it not deviated from the visual communication space. At the same time, it is necessary to repeatedly test when operating multiple optical communication links to determine if the final visual work can achieve the intended purpose.

RETRACTED

### 2.3. Process Control

In each visual communication link, the idea and behavior work together to complete a complex task. To achieve the final result of the communication, the process control connection is essential. Based on the information from the value chain and understanding of the entire project, the visual communication is controlled by various methods, which control the process of visual communication, such as planning and management of work conditions. In some cases, it ensures that the work can produce the expected results within the set time range.

Based on Figure 2, it can be seen that due to the factors involved in different visual communication tasks and the complexity of teamwork during operation, the process control links are more closely related. Compared with comprehensive ideas and visual ideas, it seems more intuitive and rationality.

### 2.4. Creative Synthesis

Creative logic refers to the rules that must be followed in the creative process to make meaningful tasks easier and more efficient. Most importantly, it is worth thinking about the creation of creative relationship logic before and after the creation. That is, creative logic not only represents the laws and relationships between the various steps and elements in the creative process but also represents how creativity must be best adapted to its creative goals and creation [16].

As shown in Figure 3, the focus of integrated creative connections in visual communication is not visual performance, but the design and arrangement of general information such as form, process, results, influence, and conveyance progress.

### 2.5. Creative Perfection

Visual creativity is the most important and simpler connection to present the final result of visual conveying. However, with the continuous change and upgrade of the market demand in the commercial world, the visual impact on the public is gradually subsidized under the initial visual fatigue. In the face of the status quo, visual ideas often need to expand and innovate with the overall creative and era background to achieve a strong visual impact, and it changes the visual level of the past, maximizing the impact of information transfer [17].

From Figure 4, it can be an intuitive understanding, and during design and operation, the links between the creative and value chains are integrated. It transfers the final design from the design language to the final product, thereby forming the full process of information communication space to meet its requirements and visual communication.

RETRACTED

## 3. Genetic Algorithm

### 3.1. Genetic Algorithm

The genetic algorithm (GA) was first proposed by John Holland in the 1970s in the USA. The algorithm was designed and proposed according to the law of evolution of organisms in nature. It is a computational model of a biological evolutionary process that simulates the mechanism of natural selection and genetics of Darwinian biological evolution and is a method to search for the optimal solution by simulating the natural evolutionary process [18]. The flow chart of the genetic algorithm is shown in Figure 5.

### 3.2. Chaos Optimization Genetic Algorithm

The principle of this algorithm is to adjust the weight and threshold in the BP neural network through a chaotic genetic algorithm (CGA) and utilize the improved output function of the BP neural network [19]. The execution process of the algorithm is as follows.

#### 3.2.1. Initial Population Chaotic Generation

For the original generator algorithm, the randomly generated initial populations will deviate from the optimal solution in algorithm training and optimization. To overcome these weaknesses, logistic mapping is used to add mixed variables to the initial population and to find the best variable optimization solution at the global level of the optimization scale using the universality of mixed motion, thus improving efficiency and accuracy. The logistics mapping is as follows:

(1) $$\begin{array}{c} \rho_{i}^{u+1}=u\rho_{i}^{\left(u\right)}\left(1-\rho_{i}^{\left(u\right)}\right). \end{array}$$

#### 3.2.2. Moderate Functions

In the actual prediction of visual communication design, the predictive results often have a certain gap with the actual identification results, and the reciprocal of the error is used as a standard fitting measurement standard. The adaptation function is as follows:

(2) $$\begin{array}{c} f=\frac{1}{G}. \end{array}$$

#### 3.2.3. Select Operation

The main basis of this work is the adaptive function. The higher the appropriate value of the individual population, the greater the possibility of being selected. Depending on the appropriateness of the policy, the probability that all individuals are selected is

(3) $$\begin{array}{c} f_{i}=\frac{l}{F_{i}},\\ p_{i}=\frac{f_{i}}{\varpi_{i=1}^{N}f_{i}}. \end{array}$$

#### 3.2.4. Cross Operation

For genetic algorithms, following the theory of populations, cross the population and the best individuals generated by the system, that is, the real cross-specific. No. *l* chromosome *α*_*l*_ and No. *kα*_*k*_ in the *i* bits are as follows:

(4) $$\begin{array}{c} \left\{\begin{array}{c} \alpha_{lj}=\alpha_{lj}\left(1-b\right)+\alpha_{ij}b,\\ \alpha_{kj}=\alpha_{ij}\left(1-b\right)+\alpha_{lj}b. \end{array}\right. \end{array}$$

RETRACTED

#### 3.2.5. Variation Operation

Species variation is a type of genetic variation, which produces a new population and then produces new individuals. Variation function in the genetic algorithm can divide a population to further expand the search. The function of selecting the individual genes is as follows:

(5) $$\begin{array}{c} f\left(m\right)=r{\left(1-\frac{m}{M_{\max}}\right)}^{2},\\ \alpha_{ij}=\left\{\begin{array}{c} \alpha_{ij}+\left(\alpha_{ij}-\alpha_{\max}\right)f\left(m\right),\;r>0.5,\\ \alpha_{ij}+\left(\alpha_{\min}-\alpha_{ij}\right)f\left(m\right),\;r\leq 0.5, \end{array}\right. \end{array}$$

where *α*_max_ and *α*_min_ represent the upper and lower limit values of *α*_*ij*_, respectively, *r* is a random number whose value interval is [0,1], *g* represents the current number of iterations, and *M*_max_ represents the upper limit value of the number of evolutions.

#### 3.2.6. Determining the Random Disturbance

(6) $$\begin{array}{c} \alpha =1-{\left(\frac{l-1}{l}\right)}^{m},\\ \Omega_{k}^{\prime }=\left(1-\alpha \right)\Omega^{\Phi }+\alpha \Omega_{k}. \end{array}$$

Here, the resulting vector is expressed by the current optimal solution on [0, 1], that is, the optimal chaotic vector. Ω_*k*_ represents the chaotic vector obtained by *k* iteration, Ω_*k*_ indicates the corresponding chaotic vector after scrambling, and *k* represents the number of iterations, where its value is [0, 1]. During the continuous iteration, the maximum value is analyzed, and *m* is an integer and is determined by the target function.

### 3.3. MIMO-SCMA System Based on Genetic Algorithm

For the MIMO-SCMA downlink system, after the final receiving antenna receives the signal, the MIMO signal is first detected, and then the next detection result is detected. MIMO detection is used to detect multidimensional signals, so it is very complicated in a single antenna system. In addition, multiple transmit antennas simultaneously increase the channel interference problem of the same channel source transmitted signal to find the difficulty of finding MIMO signals [20].

Suppose that the signal transmitted by the antenna at the base station is shown in Equation (7), and the signal received by the antenna at the user end is shown in Equation (8).

(7) $$\begin{array}{c} x=\left[{\left(x^{1}\right)}^{T},{\left(x^{2}\right)}^{T},\ldots ,{\left(x^{D_{B}}\right)}^{T}\right]\in C^{N_{B}K\times 1}, \end{array}$$

(8) $$\begin{array}{c} y=\left[{\left(y^{1}\right)}^{T},{\left(y^{2}\right)}^{T},\ldots ,{\left(y^{N_{M}}\right)}^{T}\right]\in C^{N_{M}^{K\times 1}}. \end{array}$$

The detection principles of the two types of algorithms are as follows.

RETRACTED

#### 3.3.1. ZF Detection

To detect the outgoing signal *x* from the received signal *y*, it is necessary to construct a matrix *W* satisfying WH = 1, where *H* denotes the channel parameters of the MIMO channel. In ZF detection, the construction matrix is

(9) $$\begin{array}{c} W={\left(H^{h}H\right)}^{-1}H^{h}. \end{array}$$

Therefore, the statistics of this detection method are shown in Equation (10), where *n* denotes the noise of the MIMO channel.

(10) $$\begin{array}{c} \hat{y}=Wy=x+{\left(H^{h}H\right)}^{-1}H^{h}n. \end{array}$$

#### 3.3.2. MMSE Detection Algorithm

MMSE detection can effectively eliminate the signal interference from other antennas, but it also increases the negative impact on the visual process. Low-Resolution Secondary Error (MMSE) effectively suppresses interference from other antennas while minimizing the effect of interference on detection. The principle is to create a table to minimize the squared error between the resolution and the transmitted signal. The matrix structure of the algorithm is as follows.

The judgment output is estimated as

(11) $$\begin{array}{c} \hat{y}=G_{\text{MMSE}}y=\left(H^{h}H+\partial^{2}I_{T}\right)H^{h}y. \end{array}$$

Then, the mean square error arising from its verdict is

(12) $$\begin{array}{c} \varpi_{\text{MMSE}}=E\left\{\left(\hat{y}-x\right){\left(\hat{y}-x\right)}^{h}\right\}=\partial^{2}{\left(H^{h}H+\partial^{2}I_{T}\right)}^{-1}. \end{array}$$

### 3.4. Real-Time Communication of Image Features Based on Particle Swarm Optimization

Based on the received multiframe image capability, a real-time communication method based on particle font features is used to complete the visual communication of multiframe images [21]. To complete the real-time transmission of multiframe image data, this paper uses the population particle algorithm to compute multiframe image data for real-time target vision communication; the process is as follows.

To understand the distinguishability within each range of the multiframe images, the variance formula of the log-likelihood ratio function corresponding to the premise of the variance equation is

(13) $$\begin{array}{c} {ℜ}_{ik}\left(P:e\right)=K\left[p{\left(l\right)}^{2}\right]-{\left(H\left[P\left(l\right)\right]\right)}^{2}. \end{array}$$

Within the equation, the log-likelihood ratio function is *p*(*l*), and the foreground range scale and background range scale of the multiframe image are *K*[*p*(*l*)^2^] and (*H*[*P*(*l*)])^2^, respectively, using a vector to describe the weights *N*; then,

(14) $$\begin{array}{c} N=\left[y_{1},y_{2},y_{3}\right]. \end{array}$$

The multiframe image attributes *y*_1_, *y*_2_, *y*_3_, and *M*′ are the best resolutions of *M*, which is the best resolution of the individual elements of the larger image extracted using particles. The particle swarm optimization algorithm controls *M*′ by assuming that the particles *A*,{*t*_1_, *t*_2_,…, *t*_a_} and *M* have the same size points; then, each particle has a solution *M*. The orientation of each particle in the population determines the relative proportion of the particle eigenvalues. Assuming that the dimension of *M* is *G*, the particle size is *u*′, each particle in the cluster is *l* (1 ≤ *l*′ ≤ *u*′), and the orientation of each particle at the *s*′th iteration is

(15) $$\begin{array}{c} \alpha_{l}\left(c^{\prime }\right)=\left(\alpha_{l1},\alpha_{l2},\ldots ,\alpha_{lg},\ldots ,\alpha_{lG}\right). \end{array}$$

Each particle currently collects the best fitness corresponding to the orientation of the local optimal solution:

(16) $$\begin{array}{c} W_{lr}\left(c^{\prime }\right)=\left(w_{l1},w_{l2},\ldots ,w_{lg},\ldots ,w_{IG}\right). \end{array}$$

The solution that best reflects the locally optimal solution of the particle fit is the current optimal solution of the particle population Ez. The population adjusts the current velocity and direction of each particle after several iterations, and the expression for the repetition is

(17) $$\begin{array}{c} W_{lr}\left(c^{\prime }+1\right)=W_{lr}\left(c^{\prime }\right)+x_{1}l_{1}\left(E_{lr}-\alpha_{lr}\left(c^{\prime }\right)\right)+x_{2}t_{2}\left(E_{lr}-\alpha_{lr}\left(c^{\prime }\right)\right), \end{array}$$

(18) $$\begin{array}{c} A_{lr}\left(c^{\prime }+1\right)=A_{lr}\left(c^{\prime }\right)+W_{lr}\left(c^{\prime }+1\right). \end{array}$$

In Equations (17) and (18), the learning factor is also a unique random number in the range [0, 1], and the collection rate of each particle in step c′ − 1 is the collection rate of each particle in step *W*_*lr*_(*c*′+1). The optimal solution *N*′ sought in this paper is the Ez obtained at the end of the iterative probing of all particles within the population, when each particle orientation does not have any change, and the Ez obtained after the repetitive checking of all particles in the population change to complete the visual communication of the image target features.

RETRACTED

## 4. Experiment of Introducing Genetic Algorithm into Font Design

To verify the effectiveness of the genetic algorithm in font design, this paper compares the evaluation results of different algorithm users. The number of experimental research subjects was set at 300, and 280 valid questionnaires were collected using the questionnaire method. The subjects investigated in this paper are all people who have more daily contact with words, such as students, teachers, and editors, based on their occupation, age, and the time of day they are exposed to the text as the basic information for the study. And Table 1 shows the specific information of the research subjects.

### 4.1. Experimental Process

Combined with the purpose of this paper's research, the experiment issued questionnaires to people of different occupations, and a total of 300 questionnaires were issued. 80 copies were distributed to students, 72 copies to teachers, 60 copies to editors, 48 copies to designers, and 40 copies to other people. The questionnaires were collected after completion, and a total of 280 valid questionnaires were collected. The relevant questionnaires were completed and collected, and the questionnaire data were used to analyze the font design studied in this paper and draw the corresponding conclusions.

### 4.2. Experiment Content

The experiments are mainly concerned with the impact of the design of fonts on readers' vision for the genetic algorithm, using different algorithms for the design of fonts, respectively, and transmitting different fonts to the range accessible to readers. Based on readers' feedback on fonts designed by different algorithms and different fonts designed by the same algorithm, readers' recognition and exposure to fonts are derived to compare the advantages of genetic algorithms in font design.

### 4.3. Experimental Data

In this paper, 300 readers of different occupations were selected and five different algorithms other than the genetic algorithm were used to study the amount of readers' attention to fonts and their satisfaction within 1 minute.

## 5. Results of Using Genetic Algorithm-Based Font Design

### 5.1. Amount of User's Attention at the Same Time

To test the effect of visual communication design based on a genetic algorithm on users' attention, an artificial intelligence algorithm and graph theory algorithm were used to compare with a genetic algorithm to test the amount of attention of test users at the same time. The test results are shown in Figure 6.

The results show that, according to Figure 6, the time was set to 0.9 s, 0.8 s, 0.75 s, 0.6 s, 0.45 s, and 0.3, respectively, to test the amount of user attention at the same time with different algorithms. As can be seen from the figure, the survey was conducted on 280 people who had returned the questionnaire, and at different times, the genetic algorithm always had a higher amount of user attention than the other algorithms. For example, at 0.3 seconds, the font designed by the genetic algorithm has 180 users' attention, which is much higher than other algorithms. It can also be concluded that genetic algorithm has a great advantage in the design of fonts.

RETRACTED

### 5.2. Amount of Attention of Users in Different Age Groups Based on Genetic Algorithm

To test the effect of fonts designed based on a genetic algorithm on the amount of attention of readers in different age groups, people aged 18–25, 26–30, 35–40, and 45–50 years old were selected from 300 people. The test results are shown in Figure 7.

The results show that the font designed based on the genetic algorithm has the highest attention level among those aged 18–25 years old, followed by those aged 26–30 years old, and gradually increases with increasing time; the attention level of all different age groups basically reached the highest at 60 s. It can be concluded that the font designed by the genetic algorithm is more popular among young people.

### 5.3. The Attention of Users to Design Font Type under Different Algorithms

For the attention of users caused by different algorithms on font type design, five different algorithms were used to test seven different types of designed fonts, and the test results are shown in Figure 8.

The results show that the amount of user attention to font type design according to different algorithms is tested in this paper for bold advertising fonts, English, etc., respectively. According to Figure 8, no matter which algorithm designs the font type, the attention of genetic algorithm designing fonts is higher than other algorithms, among which users pay the highest attention to advertising fonts. Based on the graphical analysis, the font type designed by the genetic algorithm better caters to the needs of the reader.

The results show that the overall user satisfaction score of different algorithms is 10. As shown in Figure 9, the average user satisfaction of genetic algorithm-based font design is 8.16, the satisfaction of artificial intelligence algorithm is 7.66, and the other algorithms had a satisfaction rate of 6.732, 7, and 6.754. The comparison shows that the fonts designed by the visual communication system based on the genetic algorithm are more satisfactory. Compared with the fonts designed by other algorithms, users' satisfaction with the fonts designed by the genetic algorithm increased by 6.52%.

## 6. Discussion

In this paper, the visual communication system is improved based on the genetic algorithm, and the problems that need attention in the system and the main construction methods are introduced. After the system was constructed, experimental tests of the genetic algorithm-based system were conducted to evaluate the practicality and effectiveness of the system, which further pointed out the direction for the optimization of the system. At the same time, the particle swarm algorithm in image transmission was used to beautify the fonts in images, so that users can get visual enjoyment when reading the paper version of the reading materials and have fun in learning, which also lays the foundation for further development of the fonts.

RETRACTED

## 7. Conclusions

This paper analyzed and composed the creative logic of visual communication based on a genetic algorithm, marked an outlook on its future development in the context of the current big data era, and drew the following research conclusions.

First, visual communication is an integrated design process that evolves with the business era and expands and updates as the business community changes. During this long process of development, certain patterns existed and changed over time between the internal links and multiple links of the visual communication process.

Secondly, the logical rules between links in the process of visual communication are a combination of sensibility and rationality and are based on the understanding and analysis of the goal of the work. The artistic inspiration and logical rigor of the visual communication process work at high speed in a seemingly chaotic but regular manner.

Thirdly, by comparing the internal links and internal logical relationships within visual communication, the whole process of visual communication can be made more clear. At the same time, research and exploration based on the concept of visual communication can complete the creative process more efficiently and accurately, thus making the final visual communication result more valuable.

Fourth, the field of visual communication can find the combination of its own logic and analysis with genetic algorithms, and then, it used big data thinking and related technology to optimize the internal aspects of visual communication and ultimately makes the value of visual communication on the existing basis to form a qualitative leap.

## Figures and Tables

**Figure 1:** Operating logic map of the link.

**Figure 2:** Logical structure diagram of the process control link.

**Figure 3:** Logical structure diagram of creative integrated links.

**Figure 4:** Visual creative link logic structure.

**Figure 5:** Genetic algorithm flow chart.

**Figure 6:** Amount of attention of users at the same time.

**Figure 7:** The amount of attention of users in different age groups.

**Figure 8:** User attention to design font types.

**Figure 9:** User satisfaction test chart.

**Table 1:** Specific information on the study population.

Profession	Number of people	Average age/year	Time to touch text/hour
Student	80	21.16	10
Teacher	72	35.3	8
Editor	60	28.69	14
Designer	48	35.16	12
Others	40	32.6	6

RETRACTED

## Data Availability

Data sharing is not applicable to this article as no datasets were generated or analyzed during the current study.
